# Effects of Different Concentrations of Ropivacaine Lumbar Plexus-Sciatic Nerve Block on Recovery from Anesthesia, Postoperative Pain and Cognitive Function in Elderly Patients with Femoral Neck Fracture

**DOI:** 10.1155/2022/4096005

**Published:** 2022-08-25

**Authors:** Pingping Cheng, Feng Ying, Yafeng Li

**Affiliations:** Department of Anesthesiology, Nanchang Hongdu Hospital of Traditional Chinese Medicine, Nanchang, Jiangxi 330000, China

## Abstract

**Objective:**

To investigate the effects of lumbar plexus-sciatic nerve block with different concentrations of ropivacaine on recovery from anesthesia, postoperative pain, and cognitive function in elderly patients with femoral neck fracture.

**Method:**

A total of 110 elderly patients with femoral neck fractures who were treated in our hospital from January 2020 to January 2022 were selected as the research objects. According to the concentration of ropivacaine, they were divided into low-, medium-, and high-concentration groups (concentrations of ropivacaine were 0.15%, 0.25%, and 0.40%, respectively), with 36, 37, and 37 cases, respectively. Extubation time, anesthesia recovery time, and hospitalization time were recorded. Cognitive symptoms were assessed by the spatial cognitive ability, working memory ability, simple computing ability, and picture recognition ability test. The pain degree of patients was assessed by visual analogue scale (VAS). The occurrence of adverse reactions in patients was recorded.

**Result:**

There was no significant difference in extubation time, anesthesia recovery time, and hospitalization time among the three groups (*P* > 0.05). The PCA time of the patients in the high-concentration group was significantly longer than that in the low- and medium-concentration groups. The dosage of sufentanil within 24 hours and total sufentanil in the high-concentration group were significantly lower than those in the low- and medium-concentration groups, and the dosage of sufentanil within 24 hours and total sufentanil in the medium-concentration group was significantly less than that in the low-concentration group (*P* < 0.05). The cognitive function score for each entry of the three groups 1 d after surgery was lower than that before surgery (*P* < 0.05); On the 1 day after operation, the cognitive function score for each entry of the patients in the low-concentration group was significantly higher than that in the middle- and high-concentration groups, and the cognitive function score for each entry in the middle-concentration group was significantly higher than that in the high-concentration group (*P* < 0.05). There was no significant difference in VAS scores between the three groups at 2 h and 8 h after surgery (*P* > 0.05); 16 h and 24 h after operation, the VAS score of patients in the high-concentration group was significantly lower than that in the low- and medium-concentration groups, and the VAS score in the medium-concentration group was significantly lower than that in the low-concentration ropivacaine group (*P* < 0.05). The incidence of adverse reactions in the high-concentration ropivacaine group was significantly higher than that in the low- and medium-concentration groups (*P* < 0.05).

**Conclusion:**

The middle concentration of ropivacaine has good analgesic and nerve block effects and has less influence on cognitive function and less adverse reactions in elderly patients.

## 1. Introduction

Femoral neck fracture is a common type of fracture in the elderly. Conventional conservative treatment of femoral neck fractures has limited therapeutic effect. The anatomical structure of the femoral neck is special, and patients often have difficulty in fracture healing and necrosis of the femoral head due to poor treatment results, resulting in poor prognosis [1, 2]. In addition, due to the weakened immunity of elderly patients, combined with other underlying diseases, low organ function, and cognitive dysfunction and abnormal circulatory and respiratory system caused by the trauma of the operation itself, the tolerance of elderly patients to anesthesia surgery is reduced. Therefore, the choice of methods and drugs is particularly important [3]. With the rapid development of regional nerve block technology, peripheral nerve block has been gradually applied to various fracture operations. Lumbar plexus-sciatic nerve block can inhibit the sensation around the hip joint, and has little effect on the functions of breathing, circulation, and urinary system, so it is widely used in clinical practice. Many studies have shown that ropivacaine is a long-acting, novel, and low-toxic amide local anesthetic, with the characteristics of separation of sensory tissue and motor tissue [4, 5]. It has been proved in clinical practice that it can achieve good analgesic effect when applied to lumbar plexus-sciatic nerve block. It is widely used in China, but its concentration has not been unified [6]. In this study, in order to reveal the optimal concentration of ropivacaine in combined lumbar plexus-sciatic nerve block provides a theoretical basis, different concentrations of ropivacaine combined lumbar plexus-sciatic nerve block anesthesia were used in elderly patients with femoral neck fractures to evaluate the efficacy and safety of different concentrations of ropivacaine in elderly patients with femoral neck fracture surgery.

## 2. Materials and Methods

### 2.1. General Information

A total of 110 elderly patients with femoral neck fracture who were treated in our hospital from January 2020 to January 2022 were selected as the research objects. According to the concentration of ropivacaine, they were divided into low-, medium-, and high-concentration groups of ropivacaine, with 36, 37, and 37 cases, respectively. The concentrations of ropivacaine in the high-, medium-, and low-concentration groups were 0.40%, 0.25%, and 0.15%, respectively. There were 15 males and 21 females in the low-concentration group, aged 68–85 years, with an average age of (73.68 ± 3.54) years; there were 13 males and 24 females in the medium-concentration group, aged 65–81 years, with an average age of (72.92 ± 3.28) years; there were 15 males and 22 females in the high-concentration group, aged 66–80 years, with an average age of (73.01 ± 3.14) years. There were no significant differences in age and gender among the three groups (*P* > 0.05). Inclusion criteria were defined as follows: ① femoral neck fracture confirmed by X-ray examination; ② age ≥ 65 years; ③ no multiple injuries and mixed injuries; ④ American Society of Anesthesiologists (ASA) III or below(ASA III: the patients also suffered from severe illness and limited physical activity, but they were able to cope with daily activities). Exclusion criteria were defined as follows: ① combined abnormal coagulation function; ② mental dysfunction, cognitive insufficiency, emotional instability; ③ no recent use of psychotropic drugs and anesthetics; ④ abnormal liver and kidney function; ⑤ allergic to local anesthetics. This study was approved by the hospital ethics committee, and the patients knew and gave informed consent.

### 2.2. Methods

All patients were made to fast and were deprived of water before surgery, and routine electrocardiogram and physical signs were monitored. Sodium lactated Ringer's solution (manufacturer: Shandong Qidu Pharmaceutical Co., Ltd., approved by H20023278, specification: 500 ml) was intravenously injected to establish venous access, and tracheal intubation was given. Anesthesia: all three groups received ropivacaine lumbar plexus-sciatic nerve block anesthesia combined with general anesthesia. A 3-4 cm port was opened in the L3-L4 space as a puncture point for lumbar plexus block, 30 ml of ropivacaine was injected (manufacturer: Hebei Yipin Pharmaceutical Co., Ltd.; National Medicine Zhunzi H20113463; Specifications: 10 ml: 75 mg), and the concentration of ropivacaine in the high-, medium-, and low-concentration groups were 0.40%, 0.25%, and 0.15%, respectively. Parasacral sciatic nerve block was performed at the puncture point 3 cm down from the middle of the line connecting the posterior superior iliac spine and the greater trochanter, and 15 mL of ropivacaine was injected. The concentration of ropivacaine in the high-, medium-, and low-concentration groups was 0.40%, 0.25%, and 0.15%, respectively. After the operation, the intravenous analgesia pump was connected, and the parameters were set as: no background dose, patient-controlled analgesia (PCA) dose was 0.05 *μ*g/kg of sufentanil citrate once, with a lock-in time of 15 min. 100 mg of intravenous flurbiprofen axetil was given as background analgesia twice a day. If the numerical rating scale (NRS) ≥ 4 points, 5 mg of paracetamol and oxycodone tablets were given orally, and if still invalid after 60 minutes, 50 mg of intramuscular injection of pethidine hydrochloride was given.

### 2.3. Observation Indicators

#### 2.3.1. Surgical Indicators

The extubation time, anesthesia recovery time, and hospitalization time of the three groups of patients were recorded.

#### 2.3.2. Cognitive Function

The tests were performed once preoperatively and once 1 day postoperatively, the whole test took 10 min and all tests were performed by the same physician. ① The method was to rotate the Chinese characters by 0, 90, 180, and 270, with 1 positive and 1 negative for each direction, to limit the patient to recognize within 10 seconds, with 4 points for each time and a total of 20 points. The higher score represented the better spatial cognitive ability of the patient. ② A word recall test was used to test working memory ability by asking the patient to recite 5 words (all words chosen were real words and not easily ambiguous) and after 2 min to recall the 5 words, 2 points were awarded for those words that could be recalled correctly [7]. ③ Simple computing skills were used to test thinking skills by doing several simple mathematical problems to test the subject's intellectual status, including adding and subtracting two single-digit numbers, subtracting two two-digit numbers, and adding and subtracting three two-digit numbers. ④The method that had pictures with bright colors and clear details needed to be described clearly within 30 s which was used to test picture recognition ability. Patients were shown 5 pictures, then 5 unseen pictures were mixed in, and patients were asked to select the pictures they had seen from 10 pictures, and 2 points were awarded for each correctly remembered picture.

#### 2.3.3. Pain Assessment

The first PCA compression time, the sufentanil dosage within 24 hours after surgery and the total sufentanil dosage during hospitalization were recorded and compared among the three groups.

Visual analogue scale (VAS) [8] was used to evaluate the pain degree of patients at 2 h, 8 h, 16 h, and 24 h after surgery. A walking scale was used, about 10 cm long, with 10 scales on one side, and the two ends are the “0” end and the “10” end, where 0 means no pain, and 10 means the most unbearable pain.

### 2.4. Statistical Processing

SPSS 21.0 statistical software was used for data analysis, and the measurement data with normal distribution and homogeneous variance were expressed in the form of ($\bar{x}$ ± *s*). The differences among multiple groups were compared using the *F*-test. The count data are expressed as rate (%). Differences between groups were tested by *χ*^2^, and *P* < 0.05 indicated statistical significance.

## 3. Results

### 3.1. Comparison of Surgical Indicators among the Three Groups of Patients

There was no significant difference in extubation time, anesthesia recovery time, and hospitalization time between the low, medium, and high-concentration groups of ropivacaine (*P* > 0.05), as shown in Table 1.

### 3.2. Comparison of Analgesic Effects among the Three Groups of Patients

The PCA time of the patients in the high-concentration group was significantly longer than that in the low- and medium-concentration groups. The dosage of sufentanil within 24 hours and total sufentanil in the high-concentration group were significantly lower than those in the low- and medium-concentration groups, and the dosage of sufentanil within 24 hours and total sufentanil in the medium-concentration group were significantly less than those in the low-concentration group (*P* < 0.05), as shown in Table 2.

### 3.3. Comparison of Postoperative Cognitive Function of the Three Groups of Patients

The cognitive function scores for each entry of patients in the low, medium, and high-concentration groups of ropivacaine 1 d after surgery were all lower than those before surgery (*P* < 0.05); on the 1 day after operation, the cognitive function scores for each entry of the patients in the low-concentration group were significantly higher than those in the medium- and high-concentration groups (*P* < 0.05); The cognitive function score for each entry in the medium-concentration group was significantly higher than that in the ropivacaine high-concentration group (*P* < 0.05), as shown in Table 3.

### 3.4. Comparison of Postoperative Pain in the Three Groups of Patients

There was no significant difference in the VAS scores between the low, medium, and high-concentration groups at 2 h and 8 h after surgery (*P* > 0.05); 16 h and 24 h after operation, the VAS score of patients in the high-concentration group was significantly lower than that in the low- and medium-concentration groups, and the VAS score in the medium-concentration group was significantly lower than that in the low-concentration group (*P* < 0.05), as shown in Table 4.

### 3.5. Comparison of Adverse Reactions in the Three Groups of Patients

The incidence of adverse reactions in the high-concentration group was significantly higher than that in the low- and medium-concentration groups (*P* < 0.05), as shown in Table 5.

## 4. Discussions

Elderly patients are often associated with medical diseases, and their physiological functions and immunity are low, which makes their tolerance to anesthesia and surgery significantly reduced. The operation itself may also lead to cognitive dysfunction and circulatory and respiratory system abnormalities in elderly patients. In order to improve the safety of surgery in elderly patients, reduce postoperative complications, and improve postoperative pain, it is necessary to strictly control the concentration of local anesthetics for nerve block [8, 9]. This study provides ideas for exploring the optimal concentration of ropivacaine in clinical practice by comparing the anesthesia effect, analgesic effect, and effect on postoperative cognition and postoperative pain of lumbar plexus-sciatic nerve block with different concentrations of ropivacaine.

The transmission of perioperative stimulation to the central system can easily lead to unstable hemodynamic fluctuations, delayed catheter removal caused by slow postoperative respiratory recovery which increases the risk of perioperative complications, and the stress response during catheter insertion and removal can also lead to hemodynamic changes, which are all important factors leading to postoperative death [10]. Therefore, the use of an appropriate amount of local anesthetic, which does not cause the patient to wake up from anesthesia and prolong the extubation time, is the key to ensuring the patient's prognosis [11]. The results of this study showed that there was no significant difference in extubation time, anesthesia recovery time, and hospitalization time between the low, medium, and high-concentration groups, indicating that the anesthesia effect of different concentrations of ropivacaine was equivalent, and there was no significant difference in the anesthetic effect of ropivacaine. Extubation time and hospitalization time were prolonged due to concentration differences, but there was no statistical difference among the three groups.

The results of this study showed that the PCA time of the patients in the high-concentration group was significantly longer than that in the low- and medium-concentration groups, and the PCA time in the medium-concentration group was significantly longer than that in the low-concentration group. It shows that the nerve block of high-concentration ropivacaine lasts longer, and the dosage of sufentanil and sufentanil within 24 hours in the high-concentration group is significantly less than that of the low- and medium-concentration groups. The dosage of sufentanil in the medium-concentration group was significantly lower than that in the ropivacaine low-concentration group because the nerve block duration of the patients in the high ropivacaine concentration group lasted longer, thus reducing the postoperative dose of opioids, suggesting that high-concentration ropivacaine has a stronger analgesic effect. In addition, the results of this study showed that there was no significant difference in the VAS scores between the three groups of patients at 2 h and 8 h after surgery, but at 16 h and 24 h after surgery, the higher the concentration of ropivacaine, the lower the VAS score of the patients, further indicating that high concentrations of ropivacaine have better analgesic effect and can effectively relieve postoperative pain. Previous studies have shown [12, 13] that low concentrations of ropivacaine have the property of blocking the separation of motor and sensory nerves, and its blocking effect also increases with the concentration of ropivacaine, which is consistent with the results of this study.

The results of this study showed that after the use of ropivacaine for nerve block, the cognitive function score for each entry of the patients was decreased, and the cognitive function score for each entry of the patients in the low-concentration group was significantly higher than that in the medium- and high-concentration groups on the 1 postoperative day, and the cognitive function score for each entry in the medium-concentration group was significantly higher than that in the high-concentration group. This indicates that the lower the concentration of ropivacaine, the smaller the impact on neurocognitive function of patients and the stimulation of surgical trauma itself on patients, especially for elderly patients with underlying diseases. High concentration of ropivacaine is more likely to cause postoperative cerebral hemodynamic changes, leading to cognitive dysfunction, and low-concentration ropivacaine reduces nerve stimulation, which may be the reason for the better recovery of cognitive function scores in patients with low-concentration ropivacaine [14]. In this study, the incidence of adverse reactions in the high-concentration ropivacaine group was significantly higher than that in the low- and medium-concentration ropivacaine groups. It may be because the low concentration of ropivacaine has little effect on the physiological and hemodynamic stability of the body, and will not affect the auxiliary muscle group and nerve function of the patient's respiratory muscles. Some studies have pointed out that low-concentration ropivacaine will not cause complete blockade of nerves because it will not significantly affect the patient's respiratory function, which improves the safety of treatment [15]. Tian et al. [16] used 0.4%, 0.5%, and 0.6% of ropivacaine for anesthesia, and found that the total adverse reaction rate of 0.6% ropivacaine was significantly higher than that of the low-concentration group. The results are consistent with this study.

In conclusion, low-concentration ropivacaine has limited nerve block effect, analgesic effect, and anesthesia maintenance time, but it has less influence on patients' neurocognitive function, fewer adverse reactions, and higher safety. Although high-concentration ropivacaine has better nerve block function and is more effective in relieving postoperative pain, high-concentration ropivacaine is accompanied by high side effects. Medium-concentration ropivacaine has good analgesic effect, can exert effective nerve block function, relieve postoperative pain, and has less impact on cognitive function and less adverse reactions in elderly patients. At the same time, it has efficacy and safety, and it is a concentration worthy of clinical promotion.

## Figures and Tables

**Table 1:** Comparison of surgical indicators among the three groups of patients (*n*, ±*s*).

Group	Extubation time (min)	Anesthesia recovery time (min)	Hospitalization time (d)
Ropivacaine low-concentration group (*n* = 36)	18.06 ± 0.78	10.75 ± 0.67	6.99 ± 0.75
Ropivacaine mid-concentration group (*n* = 37)	17.95 ± 1.23	10.96 ± 0.64	7.05 ± 0.62
Ropivacaine high-concentration group (*n* = 37)	18.22 ± 0.97	11.08 ± 0.73	7.11 ± 0.83
*F*	0.666	2.190	0.241
*P*	0.516	0.117	0.786

**Table 2:** Comparison of analgesic effects among the three groups of patients (*n*, ±*s*).

Group	First compression PCA time (h)	Sufentanil dosage within 24 hours (*μ*g)	Total sufentanil dosage (*μ*g)
Low-concentration group (*n* = 36)	9.72 ± 3.21	17.59 ± 3.52	41.36 ± 6.27
Mid-concentration group (*n* = 37)	12.35 ± 4.48	15.46 ± 3.36	35.49 ± 5.74
High-concentration group (*n* = 37)	15.25 ± 4.56	11.23 ± 3.01	22.67 ± 5.35
*F*	16.320	35.200	99.670
*P*	<0.001	<0.001	<0.001

**Table 3:** Comparison of postoperative cognitive function among the three groups of patients (*n*, ±*s*).

Group	Spatial cognitive ability (score)		Working memory ability (score)		Simple computing ability (score)		Picture recognition ability (score)	
	Preoperative	1 d after surgery	Preoperative	1 d after surgery	Preoperative	1 d after surgery	Preoperative	1 d after surgery
Low-concentration group (*n* = 36)	15.86 ± 1.22	14.52 ± 0.92	8.44 ± 1.06	7.23 ± 1.10	4.06 ± 0.63	3.56 ± 0.56	9.06 ± 0.33	8.50 ± 0.51
Mid-concentration group(*n* = 37)	15.74 ± 1.31	14.10 ± 0.84	8.37 ± 1.10	6.72 ± 0.88	4.11 ± 0.70	3.19 ± 0.88	9.05 ± 0.40	8.19 ± 0.70
High-concentration group (*n* = 37)	15.79 ± 1.34	13.65 ± 0.90	8.40 ± 1.09	6.15 ± 0.74	4.11 ± 0.77	2.76 ± 0.93	9.05 ± 0.52	7.84 ± 0.76
*F*	0.079	8.784	0.038	12.680	0.061	8.950	0.007	8.962
*P*	0.924	<0.001	0.963	<0.001	0.941	<0.001	0.993	<0.001

**Table 4:** Comparison of postoperative pain levels among the three groups of patients (*n*, ±*s*).

Group	VAS scale (score)			
	2 h after surgery	8 h after surgery	16 h after surgery	24 h after surgery
Low-concentration group (*n* = 36)	1.83 ± 0.41	1.52 ± 0.39	1.48 ± 0.36	1.34 ± 0.25
Mid-concentration group (*n* = 37)	1.82 ± 0.39	1.53 ± 0.22	1.29 ± 0.20	1.18 ± 0.28
High-concentration group (*n* = 37)	1.79 ± 0.44	1.42 ± 0.25	1.19 ± 0.15	1.02 ± 0.16
*F*	0.093	1.567	12.460	16.850
*P*	0.912	0.213	<0.001	<0.001

**Table 5:** Comparison of adverse reactions among the three groups of patients (*n*, (%)).

Group	Feverr	Feel sick and vomit	Itching	Poor sight	Dizziness	Total adverse reaction rate (%)
Low-concentration group (*n* = 36)	1	2	1	0	0	5 (13.89)
Mid-concentration group (*n* = 37)	1	3	0	1	1	6 (16.22)
High-concentration group (*n* = 37)	3	4	2	1	3	14 (37.84)
*χ * ^2^						7.305
*P*						0.026

## Data Availability

The raw data supporting the conclusion of this article will be available from the authors without undue reservation.
